The article "Application Value of Mathematical Models of Diffusion-Weighted Magnetic Resonance Imaging in Differentiating Breast Cancer Lesions" was retracted in 2023. Reasons: unreliable results or conclusions; concerns about the data; concerns about the peer review; concerns about the citations.

# Application Value of Mathematical Models of Diffusion-Weighted Magnetic Resonance Imaging in Differentiating Breast Cancer Lesions

**DOI:** 10.1155/2021/1481271

**Published:** 2021-08-28

**Authors:** Xiaolong Jiang, Chao Chen, Jie Liu, Sheng Liu

**Affiliations:** The Affiliated Nanhua Hospital, Department of Radiology, Hengyang Medical School, University of South China, Hengyang, Hunan 421001, China

## Abstract

**Objective:**

To determine the application value of the mono-exponential model, dual-exponential model, and stretched-exponential model of MRI with diffusion-weighted imaging (DWI) in breast cancer (BC) lesions.

**Methods:**

Totally 64 cases with BC admitted to our hospital between June 2019 and October 2020 were enrolled in this study. They had 71 lesions in total, including 40 benign tumor lesions (including 9 breast cyst lesions) and 31 malignant tumor lesions. After DWI examination, with normal glands as control, mono-exponential model (ADC) map, dual-exponential model (Standard-ADC) map, slow apparent diffusion coefficient (Slow-ADC) map, fast-apparent diffusion coefficient (Fast-ADC) map, and stretched-exponential model (DDC) map were processed, and corresponding values were generated. Then, the situation and significance of each parameter in breast cysts, benign breast tumor lesions, and malignant tumor lesions were analyzed.

**Results:**

The values of ADC, Standard-ADC, and DDC of breast cysts were higher than those of normal glands (all *P* < 0.05), and the values of ADC and DDC of benign breast tumor lesions were lower than those of normal glands (*P* < 0.05). In addition, malignant breast tumor lesions had lower values of ADC, Standard-ADC, Slow-ADC, and DDC and a higher Fast-ADC value compared to normal glands (all *P* < 0.05). Compared with benign tumor lesions, malignant tumor lesions had lower values of ADC, Standard-ADC, Slow-ADC, and DDC and a higher value of Fast-ADC (all *P* < 0.05). Moreover, the receiver operating characteristic (ROC) curve-based analysis revealed that all the above models could be adopted to effectively evaluate the deterioration of benign breast tumor lesions (all *P* < 0.05), and DDC value had the most significant diagnostic effect on malignant tumor lesions (*P* < 0.05).

**Conclusion:**

Both dual-exponential model and stretched-exponential model of DWI can help effectively evaluate the progression of benign breast tumors, and the stretched-exponential model is more effective in the diagnosis of malignant breast tumors. These models are of great help to the future clinical diagnosis of BC.

## 1. Introduction

Breast cancer (BC) is the most pervasive malignant tumor in women worldwide, and its incidence rate stays at a high level [1]. According to statistics, there are approximately 230,000 new cases of BC each year, showing an increasing trend [2]. Due to the insidious symptoms of early BC, most patients with it have already entered the middle or advanced stage at diagnosis [3]. This is also one of the leading causes for the unfavorable prognosis of patients with BC. In addition, advanced BC is highly likely to have distant metastasis, so the treatment of BC is more difficult [4]. One survey has showed that the 5-year survival rate of patients with late BC is only 20%–30% [5]. Clinically, early diagnosis and therapy of BC is the key to protect the life and health of patients with it [6]. However, at the current stage, the diagnostic gold standard for BC still depends on pathological biopsy. Therefore, finding a novel diagnostic scheme for BC is the difficulty to be solved in clinical research.

Imaging technologies are one of the indispensable means in the diagnosis of tumor diseases. Among them, magnetic resonance imaging (MRI) with diffusion-weighted imaging (DWI) is a relatively new concept in MRI examination. It can help judge the development and progression of diseases by stimulating molecular diffusion movement in human body with molecular heat energy and forming visual images [7]. As the only noninvasive way to detect the diffusion movement of water molecules in living tissues, DWI has been verified to be able to provide highly reliable diagnostic opinions for ultra-early cerebral ischemia injury [8]. DWI has also been found to have extremely high application value in tumor diseases such as cholesteatoma, myeloma, and BC [9–11].

The classical imaging method for DWI is spin-echo echo-planar imaging (SEEPI) whose limitation is that the imaged microstructure fails to completely present the dispersion of all water molecules [12]. In recent years, a growing number of researchers have pointed out the remarkable improvement of different DWI mathematical models such as the mono-exponential model, dual-exponential model, and stretched-exponential model in the diagnosis of diseases [13, 14]. This study analyzed the application of different imaging models in breast lesions, with the goal of finding the most suitable DWI scheme for future BC diagnosis and providing reference guidance for clinical practice.

## 2. Materials and Methods

### 2.1. Research Objects

Totally 64 cases with BC admitted to our hospital between June 2019 and October 2020 were enrolled in this study. They had 71 lesions in total, including 40 benign tumor lesions (including 9 breast cyst lesions) and 31 malignant tumor lesions. This experiment was carried out with the approval of the Ethics Committee of our hospital after obtaining informed consent forms signed by all enrolled individuals.

#### 2.1.1. Inclusion and Exclusion Criteria

The inclusion criteria were as follows: patients confirmed with BC according to MRI examination and pathological examination after admission and patients with detailed clinical data. The exclusion criteria were as follows: patients with other comorbid tumors, nervous system-associated diseases, or chronic cardiovascular or cerebrovascular diseases, patients with liver or kidney dysfunction, patients unable to communicate normally, patients allergic to drugs, patients who had received radiotherapy, chemotherapy, and surgery within half a year before admission, pregnant patients, and lactating patients.

### 2.2. Determination Means

Each patient was asked to lie in a prone position with upper limb lifted, and the bilateral mammary glands were let to naturally hang within the circle. (1) Parameters for MR plain scan were as follows: T2WI; TR: 4040 ms; TE: 50 ms; FOV: 360 mm × 360 mm; BW: 83.33 kHz; echo chain length: 14; slice thickness: 4 mm; slice gap: 1 mm; matrix: 320 × 224. (2) T2WI: TR: 500 ms; TE: the minimum one; BW: 62.5 kHz; echo chain length: 3; others were the same as those of (1). (3) Single b-value DWI: two diffusion sensitivity coefficients were selected for a single excitation spin plane echo sequence (b: 0 and 800 s/mm^2^); TR: 3600 ms; TE: the minimum one; FOV: 360 mm × 360 mm; BW: 250 kHz; others were the same as those of (1). A corresponding pseudo-color map of apparent diffusion coefficient was obtained, and the ADC value in lesions was calculated with ROI. (4) Multi-b-value DWI: 12 b values were selected (0, 10, 20, 30, 50, 100, 200, 400, 800, 1200, 2000, and 3000 s/mm^2^) and others were the same as those of (3). (5) Dynamic contrast-enhanced MR: magnetic resonance breast volume imaging technology; TR: 3.9 ms; TE: the minimum one; BW: 200 kHz; slice thickness: 1.4 mm; others were the same as those of (1). Single scan was run for 50 s, with 60-second delay between period 5 and 6.

#### 2.2.1. Image Processing

The images were processed with the Functool software, and ROI (18 mm^2^) was set under the premise of avoiding areas with cystic change, necrosis, and bleeding. With normal glands as control, mono-exponential model (ADC) map, dual-exponential model (Standard-ADC) map, slow apparent diffusion coefficient (Slow-ADC) map, fast-apparent diffusion coefficient (Fast-ADC) map, and stretched-exponential model (DDC) map were processed, and corresponding values were generated.

#### 2.2.2. Outcome Measures

We observed the differences in DWI parameters of breast cysts, benign tumor lesions, and malignant tumor lesions, analyzed the diagnostic value of each parameter for breast cancer, and explored the relationship between the parameters.

### 2.3. Statistical Analyses

SPSS22.0 software was adopted for statistical analyses of all data. GraphPad Prism 8 software was used to make all charts. All calculations were repeated three times and then averaged. The obtained data were expressed as ($\bar{x}\pm s$) and compared between groups via the independent-samples *T* test. In addition, the predictive value was analyzed using ROC curves. *P* < 0.05 suggests a remarkable difference.

## 3. Results

### 3.1. Changes in DWI Parameters of Breast Cysts

The values of ADC, Standard-ADC, and DDC of breast cysts were all higher than those of normal glands, and the differences were statistically significant (*P* < 0.05), but the values of Slow-ADC and Fast-ADC of breast cysts were not different from those of normal glands, and the differences were statistically significant (*P* < 0.05) (Figure 1).

### 3.2. Diagnostic Value of DWI for Breast Cysts

According to ROC analysis, ADC value had a sensitivity of 66.67% and a specificity of 88.89% in predicting breast cysts; Standard-ADC value had a sensitivity of 66.67% and a specificity of 100.0% in predicting breast cysts; DDC value had a sensitivity of 88.89% and a specificity of 77.78% in predicting breast cysts, and the differences were statistically significant (*P* < 0.05) (Figure 2).

### 3.3. Changes in DWI Parameters of Benign Breast Tumor Lesions

The values of ADC and DDC of benign breast tumor lesions were both lower than those of normal glands, and the differences were statistically significant (*P* < 0.05), while the values of Standard-ADC, Slow-ADC, and Fast-ADC of benign breast tumor lesions were not different from those of normal glands, and the differences were statistically significant (*P* < 0.05) (Figure 3).

### 3.4. Diagnostic Value of DWI for Benign Tumor Lesions

According to ROC analysis, ADC value had a sensitivity of 74.19% and specificity of 86.78% in predicting benign tumor lesions; DDC value had a sensitivity of 80.65% and specificity of 67.74% in predicting benign tumor lesions, and the differences were statistically significant (*P* < 0.05) (Figure 4).

### 3.5. Changes in DWI Parameters of Malignant Breast Tumor Lesions

The values of ADC, Standard-ADC, Slow-ADC, and DDC of malignant breast tumor lesions were all lower than those of normal glands, and the differences were statistically significant (*P* < 0.05), while the Fast-ADC value of malignant breast tumor lesions was higher than that of normal glands, and the differences were statistically significant (*P* < 0.05) (Figure 5).

### 3.6. Diagnostic Value of DWI for Malignant Tumors

According to ROC analysis, ADC value had a sensitivity of 67.96% and specificity of 96.77% in predicting malignant tumor lesions; Standard-ADC value had a sensitivity of 90.32% and specificity of 70.97% in predicting malignant tumor lesions; Slow-ADC value had a sensitivity of 77.42% and specificity of 87.10% in predicting malignant tumor lesions; Fast-ADC value had a sensitivity of 83.87% and specificity of 83.87% in predicting malignant tumor lesions; DDC value had a sensitivity of 87.10% and specificity of 96.77% in predicting malignant tumor lesions, and the differences were statistically significant (*P* < 0.05) (Figure 6).

### 3.7. Comparison between DWI Parameters of Benign Breast Tumor Lesions and Those of Malignant Breast Tumor Lesions

Compared with benign tumor lesions, malignant tumor lesions had lower values of ADC, Standard-ADC, Slow-ADC, and DDC and a higher value of Fast-ADC, and the differences were statistically significant (*P* < 0.05) (Figure 7).

### 3.8. Value of DWI in Predicting the Transformation of Benign Tumors into Malignant Tumors

According to ROC analysis, ADC value had a sensitivity of 64.52% and a specificity of 87.10% in predicting the transformation of benign tumors into malignant tumors; Standard-ADC value had a sensitivity of 87.10% and a specificity of 87.10% in predicting the transformation of benign tumors into malignant tumors; Slow-ADC value had a sensitivity of 87.10% and a specificity of 87.10% in predicting the transformation of benign tumors into malignant tumors; Fast-ADC value had a sensitivity of 77.42% and a specificity of 93.55% in predicting the transformation of benign tumors into malignant tumors; DDC value had a sensitivity of 93.55% and a specificity of 87.10% in predicting the transformation of benign tumors into malignant tumors, and the differences were statistically significant (*P* < 0.05) (Figure 8).

## 4. Discussion

The attenuation of diffusion signal in traditional DWI is carried out according to the formula “*S*_*b*_/*S*_0_ = exp (−bD),” but the ADC value calculated according to this formula cannot fully represent the diffusion of all water molecules in imaging [15], so the diagnosis effect of traditional DWI for breast cancer is not ideal [16]. The diffusion formula of the dual-exponential model is “S_*b*_/*S*_0_ = fast diffusion scale ADC exp (−b Standard-ADC) + (1−fast diffusion scale ADC) exp (−b Slow-ADC).” The formula realizes imaging based on the physical basis of proton pool separation of parenchymatous tissue, so it has a more detailed and comprehensive imaging effect than traditional DWI [17]. However, when there is continuous distribution and diffusion due to a large number of proton pools, the dual-exponential model is unable to realize imaging [18]. At this time, the stretched-exponential model (*S*_*b*_/*S*_0_ = exp (−b DDC) ^diffusion heterogeneity index^), a DWI model with the most standard diffusion coefficient characteristics, can not only handle the uniformity of internal structure but also fully reflect the change of diffusion index [19, 20]. At the current stage, DWI is relatively rarely applied in BC. Therefore, this study preliminarily analyzed the above DWI mathematical model to provide reference and guidance for the diagnosis of BC in the future.

In this experiment, we found for the first time that the ADC value of breast cyst increased, while the ADC value of benign and malignant tumor lesions decreased. ADC is the most direct reaction parameter of water molecule diffusion ability in tissues, and the increase of its value indicates relatively strong water molecule diffusion ability [21]. We speculate that the rise of ADC value of breast cysts may be due to the following fact: the main components in cysts are water, blood, and mucus [22], and water molecules have a large space for movement in breast cysts, so they have strong diffusion movement ability. The decrease of ADC value of tumor lesions may be due to the fact that tumor cells are the main part in tissue at this time, and the tissue is accompanied by different degrees of fibrosis and necrosis [23], so the diffusion of water molecules is limited, and the value of ADC is thus reduced. According to the observation results of the dual-exponential model, we found an increase in Standard-ADC value of breast cysts, an increase in Fast-ADC value in malignant tumors, and decreases in Standard-ADC and Slow-ADC values of malignant tumors. We infer that the above differences may be related to the following facts. the abnormal proliferation of tumor cells in BC tissue led to the increase of cell density and the decrease of extracellular space. Because of the viscosity of the cell membrane, the permeability of the cell membrane was reduced, and the diffusion of water molecules in tissue cells was thus suppressed. Moreover, increases in the density and cell composition of malignant tumors could increase the proportion of diffusion heterogeneity index [24], which directly caused the decrease of Slow-ADC. In one previous study [25], the value of Standard-ADC, as an evaluation parameter integrating values of Slow-ADC and Fast-ADC, involves the real diffusion movement of water molecules and tissue perfusion. The decrease in Standard-ADC value of malignant tumor lesions fully demonstrated that the integrity of the cell membrane of breast malignant tumors was seriously damaged, and the intracellular chromatin and organelles inhibited the transmembrane diffusion of water molecules to the inside and outside [26]. The difference in the value of DDC can also preliminarily support our above views and confirm the unstable morphology of malignant tumor lesions. As we all know, DDC value can help effectively evaluate the diffusion coefficient of continuous distribution caused by a large number of proton pools, so it is often used for the diagnosis of cerebrovascular diseases with extremely complex tissues [27]. For cases with BC accompanied by accelerated proliferation of tumor cells and a large number of new blood vessels, DDC value can also reflect the continuity of tumor space more effectively. In addition, this may be the reason why the DDC value has the most significant diagnostic effect on malignant tumor diseases.

However, because of the small number of cases enrolled in this study, it is not excluded that the statistical calculation of some results may be accidental. In addition, this study has only preliminarily analyzed the mono-exponential model, dual-exponential model, and stretched-exponential model of DWI, and there may be other models with better diagnostic effect for BC. According to the above limitations, we will make a better experimental analysis as soon as possible and make an in-depth study on the application of DWI in BC and more tumor diseases, so as to provide a more comprehensive reference for clinical practice.

## 5. Conclusion

To sum up, both dual-exponential model and stretched-exponential model of DWI can help effectively evaluate the progression of benign breast tumors, and the stretched-exponential model is more effective in the diagnosis of malignant breast tumors. These models are of great help to the future clinical diagnosis of BC.

## Figures and Tables

**Figure 1:** Changes in DWI parameters of breast cysts. (a) Comparison of ADC value. (b) Comparison of Standard-ADC value. (c) Comparison of Slow-ADC value. (d) Comparison of Fast-ADC value. (e) Comparison of DDC value. # indicates differences between the two groups.

**Figure 2:** Diagnostic value of DWI for breast cysts. (a) ROC curve of ADC value in predicting breast cysts. (b) ROC curve of Standard-ADC value in predicting breast cysts. (c) ROC curve of DDC value in predicting breast cysts.

**Figure 3:** Changes in DWI parameters of benign breast tumor lesions. (a) Comparison of ADC value. (b) Comparison of Standard-ADC value. (c) Comparison of Slow-ADC value. (d) Comparison of Fast-ADC value. (e) Comparison of DDC value. # indicates differences between the two groups.

**Figure 4:** Diagnostic value of DWI for benign tumor lesions. (a) ROC curve of ADC value in predicting benign tumor lesions. (b) ROC curve of DDC value in predicting benign tumor lesions.

**Figure 5:** Changes in DWI parameters of malignant breast tumor lesions. (a) Comparison of ADC value. (b) Comparison of Standard-ADC value. (c) Comparison of Slow-ADC value. (d) Comparison of Fast-ADC value. (e) Comparison of DDC value. # indicates differences between the two groups.

**Figure 6:** Diagnostic value of DWI for malignant tumor lesions. (a) ROC curve of ADC value in predicting malignant tumor lesions. (b) ROC curve of Standard-ADC value in predicting malignant tumor lesions. (c) ROC curve of Slow-ADC value in predicting malignant tumor lesions. (d) ROC curve of Fast-ADC value in predicting malignant tumor lesions. (e) ROC curve of DDC value in predicting malignant tumor lesions.

**Figure 7:** Comparison between DWI parameters of benign breast tumor lesions and those of malignant breast tumor lesions. (a) Comparison of ADC value. (b) Comparison of Standard-ADC value. (c) Comparison of Slow-ADC value. (d) Comparison of Fast-ADC value. (e) Comparison of DDC value. # indicates differences between the two groups.

**Figure 8:** Value of DWI in predicting the transformation of benign tumors into malignant tumors. (a) ROC curve of ADC value in predicting the transformation. (b) ROC curve of Standard-ADC value in predicting the transformation. (c) ROC curve of Slow-ADC value in predicting the transformation. (d) ROC curve of Fast-ADC value in predicting the transformation. (e) ROC curve of DDC value in predicting the transformation.

## Data Availability

The data used to support the findings of this study are available from the corresponding author upon request.
